# *Bombyx batryticatus* Cocoonase Inhibitor Separation, Purification, and Inhibitory Effect on the Proliferation of SMCC-7721 HeLa-Derived Cells

**DOI:** 10.1155/2022/4064829

**Published:** 2022-06-14

**Authors:** Houwei Wang, Lingchuan Xu, Yanling Dou, Jiachao Wang

**Affiliations:** ^1^School of Pharmacy, Shandong University of Traditional Chinese Medicine, Jinan 250355, China; ^2^School of Intelligence and Information Engineering, Shandong University of Traditional Chinese Medicine, Jinan 250355, China; ^3^School of Basic Medicine, Hebei Medical University, Shijiazhuang 050017, China

## Abstract

The present study was to isolate and purify *Bombyx batryticatus* cocoonase inhibitor (BBCI) and to evaluate its inhibitory effect on the proliferation of SMCC-7721 cells. BBCI was purified from the crude proteins of *Bombyx batryticatus* using affinity chromatography with cocoonase as the ligand, its *N*-terminal amino acid sequence was determined using the Edman degradation method, and its inhibiting activity on SMCC-7721 cell proliferation was detected in vitro using the MTT method and in vivo in tumor-bearing nude mice. The purified BBCI presented as a single band in SDS-PAGE, the molecular weight determined by time-of-flight mass spectrometry was 13,973.63 Da, and its *N*-terminal amino acid sequence was VRNKRQSNDD. BBCI was a noncompetitive cocoonase inhibitor with an average Michaelis constant of 76.50, and it inhibited cocoonase activity with an inhibition ratio of 1 : 1 (molar). BBCI could inhibit the proliferation of SMCC-7721 cells in vitro with the IC_50_ being about 260.52 *μ*g/ml within 36 h of treatment and inhibit the SMCC-7721 tumor growth in nude mice by subcutaneous injection of BBCI around the tumor, where the tumor inhibitory effect was dose dependent. BBCI did not significantly influence the spleen coefficient of the mice. In conclusion, to the best of our knowledge, the present study is the first to report that BBCI, which was purified from *Bombyx batryticatus*, was a serine proteinase inhibitor with antitumor activity.

## 1. Introduction

A wide variety of investigations conducted in small animal models or cell-based systems have reported on the efficacy of natural bioactive compounds as potential anticancer therapeutics [1–4]. The traditional Chinese medicine *Bombyx batryticatus* is the dried body of the fourth-to-fifth instar larvae of *Bombyx mori* Linnaeus infected with *Beauveria bassiana* (Bals.) Vuillant and is listed in the Pharmacopoeia of the People's Republic of China (One). *Bombyx* batryticatus has the effects of dispelling wind to relieve spasm, dispelling wind to relieve pain and resolving phlegm to relieve masses [5]. *Bombyx batryticatus* is used alone or in combination with other Chinese medicines to treat various neoplastic diseases [6]. In some areas of China, *Bombyx batryticatus* is also used as a folk medicine to treat cancer [7]. There have been some reports that *Bombyx batryticatus* has antitumor effects, for example, the inhibitory effects of the water extract of *Bombyx batryticatus* on mouse sarcoma cells [8, 9], mouse Ehrlich ascites tumor cells, and human liver cancer cells [10, 11]. The inhibitory effects of the ethanol extract of *Bombyx batryticatus* on HeLa cells [12]. The inhibitory effects of three components (ergosterol, *β*-sitosterol, and palmitic acid) of *Bombyx batryticatus* on mouse melanoma cells and human melanoma cells [13]. Rat medicated serum prepared by intragastric administration of the water decoction of *Bombyx batryticatus* can inhibit the proliferation and invasion of Hepa1-6 hepatocarcinoma cells in vitro [14].

Serine protease inhibitors are widely found in animals and plants and have been generally recognized as promising candidates for cancer treatment in the medical field [15–17]. Serine protease activity in the tumor extracellular matrix is closely related to tumor invasion and metastasis [18]. There are serine protease inhibitor receptors on the membrane of cancer cells, and the combination with the inhibitors can inhibit tumor cell infiltration and metastasis [19–22]. In addition, this inhibitor can regulate the activity of matrix serine protease, inhibit the decomposition of matrix protein by protease, repair the cell barrier, and reduce the angiogenic reaction limiting tumor cell development [23–26].

Cocoonase is a serine protease synthesized and secreted by the mandible of the silkworm moth after the pupa of the silkworm emerges into a moth. It is used to dissolve the cocoon silk and form an eclosion hole in the closed cocoon shell to help the silkworm moth emerge from the cocoon. In the preliminary work of the present study, the isolation and purification of the cocoonase from the silkworm moth and its gene cloning and expression were performed (GenBank accession no.: BAJ46146.1) [27].

The present study aimed to use affinity chromatography with cocoonase as the ligand as the primary separation method to separate and purify small-molecular-weight serine protease inhibitors from the water extract of *Bombyx batryticatus*. Its physicochemical and enzymatic properties were further studied. We found that the enzyme inhibited the proliferation of SMCC-7721 cells in vitro and in vivo, and its antitumor activity mechanism was further analyzed. To the best of our knowledge, there has been no report on the antitumor activity of the low-molecular-weight protein components of *Bombyx batryticatus*. The present study provided a theoretical basis for *Bombyx batryticatus* use in the treatment of tumorous diseases in Traditional Chinese medicine clinics.

## 2. Materials and Methods

### 2.1. Animals

A total of 60 male BALB/c mice without specific pathogens (initial body weight, 22–24 g; 6–8 weeks old) were provided by Jinan Pengyue Experimental Animal Breeding Co., Ltd. (Jinan, China) with quality certificate no. SYXK (Lu) 20170022. They were allowed to acclimate for 3 days and were raised in a specific pathogen-free environment at 22°C, 50%–60% humidity with a 12-hour light/dark cycle, and *ad libitum* access to food and water throughout the experiment. All animal treatments were conducted in strict accordance with the recommendations of the National Institutes of Health Guidelines for the Care and Use of Laboratory Animals. The experiments were approved by the Institutional Animal Care and Use Committee of Shandong University of Traditional Chinese Medicine (Jinan, China).

### 2.2. Chinese Herbal Medicine

*Bombyx batryticatus* was specially prepared by Pharmacognosy Laboratory, School of Pharmacy, Shandong University of Traditional Chinese Medicine (Jinan, China) according to the processing specifications of the People's Republic of China Pharmacopoeia [5]. Silkworms at the 2nd day of the fourth instar, which were a hybrid of Qingsong × Haoyue, were infected with the pure-bred *Beauveria bassiana* (Bals.) Vuillant strain. Routine mulberry leaf breeding was carried out. *Bombyx batryticatus* was collected and dried at 40°C in an oven.

### 2.3. Extraction and Separation of *Bombyx batryticatus* Cocoonase Inhibitor (BBCI)

According to literature [28], a paper we previously published, making slight adjustments, a total of 100 g freshly prepared *Bombyx batryticatus* was homogenized in 10-fold its volume of extraction buffer (0.05 mol/l, pH 8.0, Tris HCl) and centrifuged at 4°C (4,650 × *g*; 10 min). The supernatant was collected after rinsing off the floating solid fatty materials, and the precipitate was extracted twice. The supernatants of the three extractions were combined and then lyophilized using a lyophilizer (FD-1D-50; Shanghai Bilon Instrument Co., Ltd.) to obtain the lyophilized crude protein powder of *Bombyx batryticatus*. The powder was redissolved in an appropriate amount of extraction buffer after weighing for further extraction using the ammonium sulfate stepwise salting-out method. The precipitates from (NH_4_)_2_SO_4_ with 25, 55, and 85% degrees of saturation steps were collected and dialyzed with distilled water at 4°C for 36 h. The supernatant was lyophilized and weighed after centrifugation at 4°C (10,464 × *g*; 10 min). The inhibitory activity to cocoonase was detected, and the (NH_4_)_2_SO_4_ precipitate with the highest inhibitory activity was designated as the crude BBCI product.

### 2.4. Protein Content Determination

According to literature [29], Lowry protein assay method was used to determine the protein content with BSA (MilliporeSigma; Merck KGaA) as the standard.

### 2.5. Affinity Chromatography

Cocoonase from the *Bombyx mori* moth was selected as the affinity chromatography ligand. Cocoonase is a serine protease secreted by the silkworm moth during the emergence process. It is used to hydrolyze the apex of the cocoon to form an eclosion hole so that the silkworm moth can come out of the cocoon. As described previously [27], the cocoonase ligand was purified and prepared. Cyanogen bromide-activated Sepharose CL-4B (Pharmacia Biotech) was coupled with an appropriate amount of cocoonase to prepare the affinity carrier according to the manufacturer's instructions (2018). The crude BBCI product was dissolved in balanced buffer solution (0.05 mol/l, pH 8.0, Tris HCl) and centrifuged at 4°C (10,464 × *g*; 10 min). The supernatant was loaded into the affinity chromatography column (1.6 × 20 cm; column volume, ∼35 ml; and column bed height, 17 cm). The column was successively washed with balanced buffer solution containing 1 mol/l NaCl, distilled water, and hydrochloric acid solution (pH 2.5). The eluent of the acid solution was immediately neutralized with Tris base (2.5 mol/l), and the neutralized eluent was combined, dialyzed, and lyophilized.

### 2.6. Gel Filtration Chromatography

The lyophilized eluate from the affinity chromatography was dissolved in an appropriate amount of eluent (50 mmol/l Tris HCl buffer, pH 8.0) and applied to a Sephadex G-50 (Pharmacia Biotech) gel filtration chromatography column (1.6 × 60 cm; column volume, ∼114 ml; and column bed height, ∼56 cm). The eluent flow rate was 1 ml/min, and the inhibitory activity of the cocoonase of each elution peak was detected.

### 2.7. Fast Protein Liquid Chromatography (FPLC) Analysis

The active protein peak components of Gel filtration chromatography were further analyzed by FPLC (ÄKTA Pure; GE Healthcare Life Sciences). The Superdex 75 Increase 10/300 GL column was equilibrated with 2 column volumes of 50 mmol/l pH 8.0 Tris HCl buffer. After loading the sample, 1.2 times the column volume of the eluent was collected with 50 mmol/l Tris HCl buffer (pH 8.0) as the eluent. The protein peak was concentrated with Ultra-46K (Merck KGaA), and the cocoonase inhibition activity peak was determined. The purified sample was stored at −80°C, and SDS-PAGE was used to detect the protein purity of the activity peak in each tube [30].

### 2.8. Time-of-Flight Mass Spectrometry Analysis

A total of 10 *μ*l BBCI sample (1 mg/ml) and 10 *μ*l *α*-cyano-4-hydroxycinnamic acid (5 mg/ml; MilliporeSigma; Merck KGaA) were pipetted and mixed well. A total of 1 *μ*l mixed liquid was dropped into the deep head of the sample, vacuumed to remove the solvent, and a 4800 Plus MALDI TOF/TOF™ Analyzer (Applied Biosystems; Thermo Fisher Scientific, Inc.) was used for mass spectrometry analysis. The laser light source was a 355 nm Nd:YAG laser with an acceleration voltage of 2 kV and a positive ion reflection detection mode.

### 2.9. Analysis of the *N*-Terminal Amino Acid Sequence of BBCI

The *N*-terminal amino acid sequence of BBCI was analyzed by KangChen BioTech Co., Ltd., using the Edman degradation method with an ABI 491A amino acid sequencer (Applied Biosystems; Thermo Fisher Scientific, Inc.) [31].

### 2.10. Analysis of the Inhibitory Activity of BBCI

Cocoonase was a trypsin-like serine protease. Based on the literature [27], cocoonase activity and cocoonase inhibitory activity were detected using *N*-benzoyl-DL-arginine-4-nitroanilide hydrochloride (BAPNA; Sigma-Aldrich; Merck KGaA) as the substrate. The sample to be tested was dissolved in reaction buffer (50 mmol/l pH 8.0 Tris HCl, 10 mmol/l CaCl_2_) to prepare a series of concentrations of BBCI solutions, 14, 28, 42, 56, 70, 84, and 98 *μ*g/ml, equivalent to 1, 2, 3, 4, 5, 6, and 7 nmol/ml. A total of 1 ml of the aforementioned concentrations of BBCI solution was mixed with 2 ml cocoonase solution (2.5 nmol/ml), and then 100 *μ*l 10 mmol/l BAPNA solution was added. After maintaining at 37°C for 5 min, 0.4 ml 33% acetic acid was immediately added to terminate the reaction. The absorbance (A) at 410 nm was detected. One unit of BBCI inhibitory activity was defined as the amount of enzyme required to decrease the A410 by 0.01.

### 2.11. Kinetic Analysis of BBCI

A total of 1 ml BBCI solution (2 and 3 nmol/ml) was mixed with 2 ml cocoonase solution (60 *μ*g/ml), and then 2, 4, 6, 8, 10, 12, 14, 16, or 18 *μ*l of the substrate BAPNA solution (10 mmol/l) was added. The system was incubated at 37°C for 5 min, and the absorbance (A) was detected at 410 nm. According to the Michaelis–Menten model, the inhibitor kinetic analysis subroutine in Origin 2018 64-bit software (https://www.originlab.com/) was used to plot and calculate the Michaelis constant (*K*_*m*_), maximum velocity (*V*_max_), and inhibition constant values.

### 2.12. Cell Culture

According to literature [28], slightly adjusted, SMCC-7721 HeLa-derived cells (ATCC) were incubated in DMEM (Gibco; Thermo Fisher Scientific, Inc.), which was formulated based on the product description, containing 10% refined calf serum (Gibco; Thermo Fisher Scientific, Inc.), which was deactivated at 56°C for 30 min, 100 U/ml penicillin, and 100 *µ*g/ml streptomycin in a 5% CO_2_ atmosphere at 37°C. Cells were subcultured following trypsinization when the SMCC-7721 cells adhered to the walls of the flask.

### 2.13. Determination of In Vitro Antitumor Activity

According to literature [28], slightly adjusted, the MTT method was used to determine the inhibitory activity of BBCI against SMCC-7721 cell proliferation. SMCC-7721 cells (1 × 10^5^ cells/ml) in the logarithmic phase were inoculated into 96-well plates (100 *µ*l/well) and treated following culture for 24 h. A total of three BBCI concentrations (500, 250, and 100 *µ*g/ml) were established, and six dual wells were established for each dose. At 36 h after treatment, the culture supernatant was discarded through aspiration from the wells, and each well was washed with PBS once. Subsequently, 100 *µ*l complete DMEM and 10 *µ*l MTT solution (5 g/l), which was formulated with normal saline and sterilized through filtration with a 0.22 *µ*m filter (MilliporeSigma; Merck KGaA), was added into each well. The culture supernatant was carefully discarded from the wells after incubating for 4 h at 37°C in a saturated 5% CO_2_ atmosphere, and then 150 *µ*l DMSO was added into each well. An enzyme-labelled instrument (3550 microplate reader; Bio-Rad Laboratories, Inc.) was used to determine the absorbance at 490 nm. Cell growth inhibition rate (%) = (1 − average *A* of the treatment group)/average *A* of the control group × 100. The IC_50_ of BBCI could be calculated using SPSS software (version 13.0; SPSS, Inc.).

### 2.14. Determination of In Vivo Antitumor Activity

According to literature [28], slightly adjusted, SMCC-7721 cells in the logarithmic phase were resuspended in DMEM at a density of 1 × 10^6^ cells/ml. Cell suspension (0.1 ml) was subcutaneously (SC) injected into the back of six BALB/C-nu mice. After 20 days, the nude mice were anesthetized by intraperitoneal injection of pentobarbital at a dose of 80 mg/kg, and the tumor was dissected after 15 min. The dissected mice were euthanized with CO_2_ at a volume displacement rate of 30%·vol/min for 5 min. The maximum tumor diameter obtained in the present study before transplant was <15 mm, and the well-grown tumor tissues were selected and cut into 1 mm^3^ sections weighing ∼40 mg. One section of the tumor tissue was transplanted into the left axilla of each nude mouse. After ∼1 week, the tumor-bearing nude mice with good tumor growth were randomly divided into five groups, with 10 mice in each group: the control group (SC injection of normal saline at 10 ml/kg once daily); the 5-fluorouracil (5-Fu) group (SC injection of 5-Fu around the tumor at 20 mg/kg once every 2 days); and the BBCI groups (SC injection of BBCI at 50, 25, and 12.5 mg/kg once daily). After 14 days of continuous administration, the mice were weighed and then euthanized with CO_2_ at a volume displacement rate of 30%·vol/min for 5 min. The tumor weights were compared among the groups, and the tumor inhibition rate was calculated. The spleen was collected and weighed to calculate the spleen coefficient according to the following formula: spleen coefficient = 10 × spleen weight (mg)/body weight (g).

### 2.15. Statistical Analysis

The data are presented as the mean ± standard error of the mean of ten animals per group and were analyzed using the SPSS package for Windows (version 19.0; SPSS, Inc., Chicago, IL, USA). Statistical analysis of the data was performed with Student's *t*-test and analysis of variance. *P* < 0.05 was considered to indicate a statistically significant difference.

## 3. Results

### 3.1. BBCI Extraction and Separation

The freshly prepared *Bombyx batryticatus* was cut, ground, homogenized, aqueously extracted, and lyophilized to obtain a water-soluble lyophilized powder. (NH_4_)_2_SO_4_ precipitates of the lyophilized powder (5,000 mg) at all levels were obtained by further using the stepwise salting-out method. The results in Table 1 indicated that total protein recovery of the precipitates was 34.64%, the 25% (NH_4_)_2_SO_4_ solution precipitated the least amount of protein, which exhibited weak specific inhibitory activity (0.21 U.mg^−1^), and the cocoonase inhibitor activities were mainly concentrated in the 55 and 85% (NH_4_)_2_SO_4_ precipitates; however, the specific inhibitory activity of the latter (2.07 U.mg^−1^) was 1.43 times that of the former (1.45 U.mg^−1^), which was similar to that of total (NH_4_)_2_SO_4_ precipitate (1.40 U.mg^−1^). Therefore, the 85% (NH_4_)_2_SO_4_ precipitate was designated as the crude cocoonase inhibitor, the inhibition recovery of which was 33.84%, and protein content was 442.79 mg, accounting for 12.68% of the total protein.

### 3.2. BBCI Purification

A total of 300 mg of the crude BBCI product was subjected to cocoonase-Sepharose 4B affinity chromatography, and two protein peaks formed (*A*_280 nm_; Figure 1(a) (A)). The first peak was between collection tubes 8 and 15, which was a salt elution peak exhibiting no BBCI activity, and the second peak was between tubes 25 and 30, which was a significant BBCI activity affinity adsorption peak that was further separated using Sephadex G-50. The results in Figure 1(a) (B) revealed that the main protein peak was between collection tubes 21 and 25, and this exhibited cocoonase inhibitory activity. There were four small contaminated protein peaks between collection tubes 5 and 20 in front of the main protein peak, all of which had no BBCI activity. The components in tubes 22–24 of the main protein peak were analyzed by 12% SDS-PAGE purity analysis, showing a single protein band, and the estimated purity was >90%. The eluents in tubes 22–24 following repeated sample loading were combined and further analyzed by FPLC. The data in Figure 1(c) demonstrated that the main peak of the protein appeared between 25 and 30 min of elution time. The main peak components were combined and collected to obtain purified BBCI. The results in Figure 1(b) revealed that the crude BBCI protein had numerous bands and a complex composition, further affinity chromatography removed the majority of the hybrid proteins and left clear main bands, and more uniform main bands of BBCI were obtained following gel filtration and FPLC, with an apparent relative molecular weight of ∼14 kDa. Time-of-flight mass spectrometry (Figure 1(d)) indicated that the BBCI molecular mass was 13,973.63 Da.

The activity recovery during each purification step is listed in Table 2. Following affinity chromatography, the specific inhibitory activity was increased 9.30-fold, and this was the key step of BBCI purification. The Sephadex G-50 separation further increased the specific inhibitory activity 1.32 times and produced a homogenous component. The activity recovery was 24.40% and 6.02-fold purified RPTI was obtained. Although the purification factor of the FPLC step was not significantly improved, the purity of BBCI was further improved to meet the requirements of *N*-terminal amino acid sequencing analysis. Using three-step chromatographic separation, 13.01-fold purified BBCI was obtained, and the activity recovery was 86.26%.

### 3.3. *N*-Terminal Amino Acid Sequence and Homology

The BBCI *N*-terminal amino acid sequence was determined following SDS-PAGE and transmembrane filtration. In the present study, the first 10 amino acid residues at the *N*-terminal of BBCI were 1-VRNKRQSNDD-10. The BLASTp program was used to search the nonredundant protein sequences (nr) database (https://blast.ncbi.nlm.nih.gov/Blast.cgi), and the *E* value range was set to 0–100. A total of six proteins with 100% similarity were retrieved (Table 3), and a phylogenetic tree with Grishin (protein) as the distance was established using the Fast Minimum Evolution method. The results in Table 3 demonstrated that BBCI was highly homologous with a *Bombyx mori* protease inhibitor (NP_001040294.1), a wild silkworm uncharacterized protein (XP_028028609.1) and a flavobacterium protein; however, they were not the same protein due to their molecular weights being different. To the best of our knowledge, the present study was the first report that BBCI was isolated and purified from the traditional Chinese medicine *Bombyx batryticatus*.

### 3.4. Inhibitory Effect and Kinetics Analysis of BBCI on Cocoonase Activity

The inhibitory activity of BBCI on silkworm cocoonase was detected. For 0–5 nM BBCI, the cocoonase inhibition activity had a good linear association with the concentration of BBCI in the reaction system containing 5 nM cocoonase (Figure 2(a)). The linear regression equation was *Y* = −1.397*x* + 99.241 (*R*^2^ = 0.999). To completely inhibit 5 nM cocoonase, 5.07 nM BBCI was required, the molar inhibition ratio was ∼1 : 1, and the mass inhibition ratio was ∼1 : 1.71 between BBCI and cocoonase.

Origin 2018 software was used for the kinetic analysis of the inhibitory activity, and the *K*_*m*_ and *V*_max_ values were calculated using the Michaelis–Menten model. The data in Figure 2(b) revealed that the *K*_*m*_ values of the three BBCI concentrations (0, 2, and 3 nM) were 76.76, 76.40, and 76.35, which were similar, and the *V*_max_ values were 46.50, 27.76, and 18.53, respectively, which decreased with the increase of BBCI content. Therefore, BBCI was a noncompetitive inhibitor of cocoonase.

### 3.5. Inhibitory Effect of BBCI on SMCC-7721 Cell Proliferation In Vitro

SMCC-7721 cells were administered with BBCI after 24 h of adherent growth, and the absorbance at 490 nm of each culture well was measured using the MTT method after 36 h of administration. BBCI markedly inhibited the proliferation of SMCC-7721 cells and the inhibition was concentration dependent (Table 4). The IC_50_ of BBCI calculated using logistic regression was 260.52 *µ*g.ml^−1^ within 36 h after treatment.

The SMCC-7721 cells were treated with 500 *µ*g.ml^−1^ BBCI (Figure 3). After 36 h of administration, the SMCC-7721 cells in the BBCI group were reduced in number compared with those of the control group, with numerous suspended cells being dead, and the cells were less shrunken with less fission, with cells exhibiting nuclear pyknosis and a rough cytoplasm. The control cells had regular shapes and good adherent growth.

### 3.6. Activity of BBCI against SMCC-7721 Cells In Vivo

Subcutaneous BBCI administration around the tumor markedly inhibited the growth of the transplanted SMCC-7721 cells with 5-Fu as the positive control drug, and the inhibition was dose dependent (Table 5). The tumor inhibition effect in the low-dose group was not significantly different from that in the control group, while those of the medium-dose and high-dose BBCI groups and the 5-Fu positive control group were markedly increased compared with that of the control group. There was no significant difference in the tumor inhibition rate between the BBCI medium-dose group and the 5-Fu group, while that of the BBCI high-dose group was higher than that of the 5-Fu group. Each dose of BBCI was not observed to have a significant effect on the spleen coefficient of the nude mice.

## 4. Discussion

The theory of traditional Chinese medicine suggests that the fickleness of “internal wind” is one of the key pathogeneses of cancer metastasis [32]. *Bombyx batryticatus* has the effect of extinguishing and expelling wind in traditional Chinese medicine clinic [5]. There have been reports on the antitumor effects of “wind medicine” [33–35], and a number of studies on the antitumor components and mechanism of *Bombyx batryticatus* [6–14], but no reports on the antitumor small-molecule active protein of *Bombyx batryticatus*. A protein component with cocoonase inhibitory activity of *Bombyx batryticatus* was isolated in previous research, and it was hypothesized that this was closely related to the antitumor activity of *Bombyx batryticatus*. Therefore, BBCI was further purified from the 85% ammonium sulfate precipitate of the *Bombyx batryticatus* crude protein by affinity chromatography with cocoonase as a ligand, Sephadex G-50 gel filtration chromatography and FPLC in sequence. The purified BBCI exhibited a single band in SDS-PAGE and a single symmetrical chromatographic main peak in FPLC. The inhibitory activity kinetics and the effects of BBCI on SMCC-7721 cell proliferation *in vitro* and *in vivo* were further analyzed to lay a foundation for the antitumor clinical application of *Bombyx batryticatus* and for the research and development of BBCI as a novel anticancer drug.

Affinity chromatography with cocoonase as the ligand was the technical core for the purification of BBCI. The cocoonase ligand was derived from a serine protease synthesized and secreted by the silkworm moth during the emergence process. The purified BBCI was a serine protease inhibitor. In affinity chromatography, it was necessary to incubate the loaded chromatographic column at 37°C for 1–1.5 h in order to hydrolyze and remove the substrate protein nonspecifically bound to the affinity ligand; then, the column was washed with 1 mol.l^−1^ NaCl solution to remove most of the impurity proteins that were nonspecifically bound to the gel medium and finally washed with a hydrochloric acid solution (pH 2–3) to obtain BBCI with a small amount of impurities.

In Sephadex G-50 gel filtration chromatography, the main active peak of BBCI was between the 20th and 25th collection tubes; however, there was a small-impurity protein peak in front of the main active peak that was not completely separated from the main peak. In order to ensure the BBCI purity, only the collection solutions of tubes 23–25 were combined together for the subsequent FPLC analysis. Using the ABI-491A amino acid sequencer to sequence according to the Edman degradation method required high protein purity. In order to ensure successful sequencing, the main peak collection solution of FPLC was subjected to PAGE and then electrotransferred to the PVDF membrane, and the main band on the membrane was cut off for sequencing analysis. The first 10 amino acid sequence of the *N*-terminal of BBCI was determined as VRNKRQSNDD.

According to the homology comparison results using the BLASTp program to search the nr database and the phylogenetic tree, BBCI is highly homologous to a precursor of the silkworm moth protease inhibitor (NP_001040294.1), of which the 21–30 amino acid sequence is exactly the same as the 1–10 sequence of BBCI. According to the results of large-scale full-length cDNA sequencing of silkworm by Suetsugu et al. [36], NP_001040294.1 contains 148 amino acid residues, and the molecular weight calculated from the 21st amino acid residue is exactly the same as that of BBCI determined by time-of-flight mass spectrometry, which is 13,973.63 Da. It can be concluded that BBCI is a serine protease inhibitor derived from the NP_001040294.1 protein deleted from the *N*-terminal 20 amino acid residues, which contains 128 amino acid residues with an isoelectric point of 8.01. The full-length amino acid sequence and cDNA coding sequence of BBCI predicted according to NP_001040294.1 were summarized in Table 6. To the best of our knowledge, this is the first report to describe BBCI isolation and purification from the traditional Chinese medicine *Bombyx batryticatus*.

BBCI had an inhibitory effect on the proliferation of SMCC-7721 cells in vitro and the tumor growth in tumor-bearing nude mice, and the inhibition rate showed a linear dose effect. Therefore, BBCI was a serine protease inhibitor with antitumor activity in *Bombyx batryticatus*.

The degradation of the tumor extracellular matrix barrier is the key in the process of tumor cell proliferation and infiltration, which is closely related to serine protease activity in the matrix [22]. It was hypothesized that BBCI could bind to the serine protease inhibitor receptors on the SMCC-7721 cell membrane, inhibit matrix protease activity, and affect the infiltration and diffusion process of tumor cells by blocking the degradation of the extracellular matrix barrier so as to have an inhibitory effect on the proliferation of SMCC-7721 cells in vitro and in vivo [37–40].

The inhibitory effect of BBCI on the proliferation of SMCC-7721 cells in vivo and in vitro revealed a good prospect for the development of antitumor drugs. However, the target and mechanism of BBCI directly inhibiting and blocking the metastasis and invasion of SMCC-7721 cells need to be further clarified. According to new landscapes and horizons in carcinoma therapy [41, 42], the next step of this research is to study the effect of BBCI on tumor-related signaling pathways to explore its antitumor mechanism in depth to demonstrate the feasibility of BBCI for antitumor clinical applications.

## 5. Conclusions

To the best of our knowledge, the present study is the first to report that BBCI was a serine proteinase inhibitor with antitumor activity. BBCI was separated and purified from an 85% (NH_4_)_2_SO_4_ precipitate of the crude protein extract of *Bombyx batryticatus* using affinity chromatography with cocoonase as the ligand. Its molecular weight was 13,973.63 Da, and its *N*-terminal amino acid sequence was VRNKRQSNDD. BBCI was a noncompetitive cocoonase inhibitor with an average Michaelis constant of 76.50, and it inhibited cocoonase activity with an inhibition ratio of 1 : 1 (molar). BBCI could inhibit the proliferation of SMCC-7721 cells in vitro and in vivo in tumor-bearing nude mice.

## Figures and Tables

**Figure 1:** Separation, purification, electrophoresis, and mass spectrometry of BBCI. (a) A Sepharose 4B cocoonase-affinity chromatography. B Sephadex G-50 gel filtration chromatography. (b) SDS-PAGE. Lane M, molecular weight markers (from top to bottom, 250, 150, 100, 70, 50, 40, 35, 25, 20, 15, and 10 kDa); Lanes 1–4, BBCI crude protein (the loading volume was 25, 20, 15, and 10 *μ*l); Lanes 5 and 6, affinity chromatography; Lane 7, gel filtration chromatography; and Lane 8, FPLC. (c) FPLC (Superdex 75 Increase 10/300 GL). (d) Time-of-flight mass spectrometry. BBCI: *Bombyx batryticatus* cocoonase inhibitor; FPLC: fast protein liquid chromatography; and OD: optical density.

**Figure 2:** Detection and kinetic analysis of the inhibitory activity of BBCI on silkworm cocoonase. (a) Detection of inhibitory activity. Following the addition of 1, 2, 3, 4, 5, 6, or 7 nM BBCI to the reaction system containing 5 nM (120 *μ*g) cocoonase and 1 *μ*M substrate BAPNA, respectively, *A*_410_ was measured. Taking the content of BBCI as the abscissa, and the average value of the remaining activity of cocoonase (*A*_BBCI_/*A*_control_ × 100%) of the three repeated experiments as the ordinate, the graph was drawn using Origin 2018 software. (b) Kinetic analysis. Following the addition of 20, 40, 60, 80, 100, 120, 140, 160, or 180 nM BAPNA to the reaction system containing 5 nM (120 *μ*g) cocoonase and 2 or 3 nM BBCI, respectively, *A*_410_ was measured. Taking the substrate BAPNA concentrations as the abscissa, and the average of the reaction speed *V* (*V* = 2.58 × 10^−5^*A*_410_) of three repeated experiments as the ordinate, the Michaelis–Menten model was used for mapping using Origin 2018 software. *A*_410_: light absorption value at 410 nm; BBCI: *Bombyx batryticatus* cocoonase inhibitor.

**Figure 3:** Effect of BBCI on SMCC-7721 cell morphology (magnification, ×100). (a) Control. (b) BBCI treatment (500 *µ*g.ml^−1^ BBCI; 36 h after addition to the cells). BBCI: *Bombyx batryticatus* cocoonase inhibitor.

**Table 1:** Isolation of BBCI crude protein by salt fractionation with (NH_4_)_2_SO_4_ and determination of its inhibitory activity.

Component	Protein content (mg)	Inhibitoryactivity (U)	Specific inhibitoryactivity (U.mg^−1^)	Inhibitionrecovery (%)	Proteinrecovery (%)
Total protein	3492.75	2711.26	0.78	100.00	100
25% (NH_4_)_2_SO_4_ precipitate	275.68	57.83	0.21	2.13	7.89
55% (NH_4_)_2_SO_4_ precipitate	491.45	713.43	1.45	26.31	14.07
85% (NH_4_)_2_SO_4_ precipitate	442.79	917.39	2.07	33.84	12.68
Total (NH_4_)_2_SO_4_ precipitate	1209.92	1688.65	1.40	62.28	34.64

BBCI: *Bombyx batryticatus* cocoonase inhibitor.

**Table 2:** Purification steps of BBCI.

Purification step	Protein content (mg)	Inhibition activity (IU)	Inhibition recovery (%)	Specific inhibition activity (U/mg)
85% (NH_4_)_2_ SO_4_ precipitate	300.00	621.59	100	2.07
Affinity chromatography	29.29	563.58	90.67	19.24
Sephadex G-50 gel filtration	21.38	541.33	87.09	25.32
FPLC (Superdex 75 Inc., 10/300 GL)	19.91	536.18	86.26	26.93

BBCI: *Bombyx batryticatus* cocoonase inhibitor.

**Table 3:** BLASTp similarity of the BBCI *N*-terminal amino acid sequence (*E* value 0–100).

Accession	Scientific name	Total score	*E* value	Per. ident (%)	Sequence
Query	*Bombyx batryticatus*	100	0	100.00	1 VRNKRQSNDD10
XP_028028609.1	*Bombyx mandarina*	35.4	0.53	100.00	21 VRNKRQSNDD 30
NP_001040294.1	*Bombyx mori*	35.4	0.55	100.00	21 VRNKRQSNDD 30
OYU82547.1	*Flavobacterium* sp. BFFFF2	32	8.9	100.00	114 VRNKRQSND 122
XP_017783957.1	*Nicrophorus vespilloides*	29.9	50	88.89	23 IRNKRQSND 31
KAF2887618.1	*Ignelater luminosus*	29.9	51	88.89	96 RNKRQANDD 104
XP_028400913.1	*Dendronephthya gigantea*	29.1	98	100.00	636 NKRQSNDD 643

BBCI: *Bombyx batryticatus* cocoonase inhibitor.

**Table 4:** Inhibitory effect of BBCI on the in vitro proliferation of SMCC-7721 cells.

Group	Concentration (*μ*g.mL^−1^)	Absorbance (*A*)	Inhibition rate (%)
Control	0	0.697 ± 0.017	—
BBCI	100.00	0.531 ± 0.034^*∗∗*^	24
	250.00	0.389 ± 0.029^*∗∗*^	44
	500.00	0.195 ± 0.025^*∗∗*^	72

Absorbance values are the mean ± SD, *n* = 10. ^*∗∗*^*P* < 0.01, compared with the control (0 *µ*g.ml^−1^) group. BBCI: *Bombyx batryticatus* cocoonase inhibitor.

**Table 5:** Tumor inhibition rate of BBCI on SMCC-7721 cells in tumor-bearing mice and the spleen coefficient.

Group	Dose (mg.kg^−1^)	Tumor weight (g)	Tumor inhibition rate (%)	Spleen coefficient (mg/g)
Control	0	0.38 ± 0.19	0	5.27
5-Fu	20.00	0.29 ± 0.16^*∗*^	23.68	5.18
BBCI	12.50	0.35 ± 0.14	9.68	5.36
	25.00	0.27 ± 0.11^*∗*^	31.43	5.63
	50.00	0.23 ± 0.09^*∗*^^,a^	55.56	5.44

Conducted in triplicate. Tumor weight and spleen coefficient values are the mean ± SD. ^*∗*^*P* < 0.01, compared with the control group. ^a^*P* < 0.05, compared with the positive control group. BBCI: *Bombyx batryticatus* cocoonase inhibitor.

**Table 6:** BBCI amino acid sequence and its cDNA coding sequence.

gta	agg	aac	aag	cgt	cag	tcg	aat	gat	gat	gat	gac	gtt	ctc	gat	gac
*V*	*R*	*N*	*K*	*R*	*Q*	*S*	*N*	*D*	*D*	*D*	*D*	*V*	*L*	*D*	*D*
cgc	tat	ggc	tgg	gag	ctt	acc	acc	cgg	cct	cca	agg	cag	ttc	cct	ggg
*R*	*Y*	*G*	*W*	*E*	*L*	*T*	*T*	*R*	*P*	*P*	*R*	*Q*	*F*	*P*	*G*
caa	gga	ttt	ttc	ccc	ggt	cta	ttc	ccc	ggc	cag	ggt	cag	ttc	cca	gga
*Q*	*G*	*F*	*F*	*P*	*G*	*L*	*F*	*P*	*G*	*Q*	*G*	*Q*	*F*	*P*	*G*
caa	cag	caa	cgt	tta	act	acg	act	cgg	gct	ccc	aac	aat	ctg	ggc	acc
*Q*	*Q*	*Q*	*R*	*L*	*T*	*T*	*T*	*R*	*A*	*P*	*N*	*N*	*L*	*G*	*T*
acc	aca	atg	tcg	cct	gca	att	caa	caa	tgc	att	cgt	agc	tgc	cca	gta
*T*	*T*	*M*	*S*	*P*	*A*	*I*	*Q*	*Q*	*C*	*I*	*R*	*S*	*C*	*P*	*V*
acc	gct	gag	tac	aat	cca	gtt	tgt	ggc	act	gat	aat	ata	act	tac	aat
*T*	*A*	*E*	*Y*	*N*	*P*	*V*	*C*	*G*	*T*	*D*	*N*	*I*	*T*	*Y*	*N*
aac	cct	gga	agg	ttg	acg	tgt	gct	cag	gcg	tgt	gga	atc	aat	gtc	agc
*N*	*P*	*G*	*R*	*L*	*T*	*C*	*A*	*Q*	*A*	*C*	*G*	*I*	*N*	*V*	*S*
gtt	ctc	cga	tcc	ctg	cct	tgc	ccc	act	gct	aca	caa	gct	cct	acc	agc
*V*	*L*	*R*	*S*	*L*	*P*	*C*	*P*	*T*	*A*	*T*	*Q*	*A*	*P*	*T*	*S*

BBCI: *Bombyx batryticatus* cocoonase inhibitor.

## Data Availability

The data used or analyzed during the current study are available from the corresponding author upon reasonable request.

## Abbreviations

BBCI: *Bombyx Batryticatus* cocoonase inhibitor.
